The article "Comparing the Effect of Dipeptidyl-Peptidase 4 Inhibitors and Sulfonylureas on Albuminuria in Patients with Newly Diagnosed Type 2 Diabetes Mellitus: A Prospective Open-Label Study" was published in 2019. Journal: J Clin Med.

# Comparing the Effect of Dipeptidyl-Peptidase 4 Inhibitors and Sulfonylureas on Albuminuria in Patients with Newly Diagnosed Type 2 Diabetes Mellitus: A Prospective Open-Label Study

**DOI:** 10.3390/jcm8101715

**Published:** 2019-10-17

**Authors:** Po-Chung Cheng, Shang-Ren Hsu, Jeng-Fu Kuo, Yun-Chung Cheng, Yu-Hsiu Liu, Shih-Te Tu

**Affiliations:** 1 Division of Endocrinology and Metabolism, Department of Internal Medicine, Changhua Christian Hospital, 135 Nanxiao Street., Changhua City, Changhua County 500, Taiwan; 180459@cch.org.tw (P.-C.C.); 67781@cch.org.tw (S.-R.H.); 103348@cch.org.tw (J.-F.K.); 2 Department of Radiology, Taichung Veterans General Hospital, Taichung Veterans General Hospital, Section 4, No. 1650, Taiwan Boulevard, Taichung, Taiwan; iancheng@vghtc.gov.tw; 3 Department of Accounting and Information Systems, National Taichung University of Science and Technology, 129 San Min Road., Taichung, Taiwan; graceliu@nutc.edu.tw

**Keywords:** proteinuria, diabetes mellitus, dipeptidyl-peptidase 4 inhibitors, sulfonylureas

## Abstract

Diabetic kidney disease (DKD) leads to substantial morbidity in patients with type 2 diabetes mellitus (T2DM). Evidence suggests that antidiabetic drug dipeptidyl-peptidase 4 (DPP-4) inhibitors may be able to attenuate albuminuria, whereas the influence of sulfonylureas on albuminuria remains unclear. This prospective open-label study investigated the effect of DPP-4 inhibitors and sulfonylureas on urinary albumin excretion, which is a marker of renal microvascular abnormality. A total of 101 participants with newly diagnosed T2DM were enrolled. In addition to metformin therapy, 45 patients were assigned to receive DPP-4 inhibitors and 56 to receive sulfonylureas. Urinary albumin-to-creatinine ratio (ACR) was significantly reduced in recipients of DPP-4 inhibitors after 24 weeks (29.2 µg/mg creatinine vs. 14.9 µg/mg creatinine, *P* < 0.001), whereas urinary ACR was not significantly changed by sulfonylureas (39.9 µg/mg creatinine vs. 43.2 µg/mg creatinine, *P* = 0.641). The effect on albuminuria occurred even though both treatment groups had a similar change in serum glycated hemoglobin A_1c_ (−1.87 % vs.−2.40 %, *P* = 0.250). Therefore, in diabetic patients the addition of DPP-4 inhibitors lowered urinary albumin excretion compared to sulfonylureas, and attenuation of albuminuria may be a consideration when choosing between antidiabetic medications.

## 1. Introduction

Diabetic kidney disease (DKD) occurs in up to 40% of patients with type 2 diabetes mellitus (T2DM) [1]. DKD leads to substantial morbidity and reduces quality of life in affected patients [2] and chronic hyperglycemia in the context of T2DM leads to microvascular injury in the diabetic kidney [3]. Current evidence suggests that clinical interventions targeting plasma glucose, body weight, and blood pressure can attenuate the development of DKD [4]. 

The article "Comparing the Effect of Dipeptidyl-Peptidase 4 Inhibitors and Sulfonylureas on Albuminuria in Patients with Newly Diagnosed Type 2 Diabetes Mellitus: A Prospective Open-Label Study" was published in 2019. Journal: J Clin Med.

Oral antidiabetic drugs such as dipeptidyl-peptidase 4 (DPP-4) inhibitors and sulfonylureas are extensively used in the treatment of T2DM. Although both DPP-4 inhibitors and sulfonylureas effectively lower plasma glucose levels, there may be differences in their effect on the diabetic kidney. Importantly, clinical evidence has suggested that DPP-4 inhibitors may be able to attenuate the progression of albuminuria in patients with T2DM [5,6]. In contrast, there is insufficient information regarding the effect of sulfonylureas on DKD. However, sulfonylureas are associated with weight gain and heart dysfunction [7], both of which may worsen albuminuria in diabetic patients. 

Considering that both DPP-4 inhibitors and sulfonylureas have a distinct effect on body weight and blood pressure, we hypothesized that these medications may influence the diabetic kidney differently. This study investigated the effect of DPP-4 inhibitors and sulfonylureas on urinary albumin excretion, a marker of renal microvascular abnormality, in patients with newly diagnosed T2DM. Moreover, the effect of these medications on clinical variables including body weight, serum glycated hemoglobin A_1c_ (HbA_1c_), and systolic blood pressure were examined.

## 2. Materials and Methods

### 2.1. Participant Selection

In this prospective study, diabetic patients who visited the Endocrinology clinic between March 2016 and February 2018 were screened for eligibility. Inclusion criteria were patients exceeding 20 years of age, with newly diagnosed T2DM, who had yet to receive antidiabetic medications. Exclusion criteria were patients with non-diabetic kidney disease, congenital kidney abnormalities, or end-stage renal disease. Moreover, patients receiving angiotensin-converting enzyme inhibitors (ACEI) or angiotensin receptor blockers (ARB) were ineligible because these medications can modify urinary albumin excretion.

### 2.2. Study Protocol

Demographic information, including age, sex, and systolic blood pressure, was recorded at the initial clinic visit. In accordance with the recommendation by the American Diabetes Association to prescribe metformin to all patients with T2DM in the absence of contraindications [5], participants received 1000 mg of metformin therapy at the beginning of the study. Subsequently, patients were assigned to receive either the DPP-4 inhibitor Vildagliptin 50 mg twice daily or the sulfonylurea Glimepiride 2 mg twice daily. Treatment allocation was made by a committee of endocrinologists to match participants in the treatment groups by age, body weight, serum HbA_1c_, urinary albumin-to-creatinine ratio (ACR), and serum creatinine. Both the investigators and the participants were informed of the treatment allocation. Participants subsequently received standard clinical care, including medical nutrition therapy and diabetes educator consultation, in accordance with current diabetes management guidelines [5].

The article "Comparing the Effect of Dipeptidyl-Peptidase 4 Inhibitors and Sulfonylureas on Albuminuria in Patients with Newly Diagnosed Type 2 Diabetes Mellitus: A Prospective Open-Label Study" was published in 2019. Journal: J Clin Med.

### 2.3. Laboratory Methods

At the initial clinic visit, participants received blood tests for serum HbA_1c_, serum creatinine, serum alanine transferase, and plasma lipid profile after a 12-hour fast. Blood tests for these clinical variables were repeated after 24 weeks of pharmacologic treatment. Blood samples were delivered to the clinical laboratory within one hour of venous sampling and assayed by Beckman Coulter UniCel DXC 800 Synchron™ Clinical Systems (Beckman Coulter, Brea, USA). The analytical precision was within 1.7 mg/dL for high-density lipoprotein cholesterol, within 3.0 mg/dL for low-density lipoprotein cholesterol, within 7.5 mg/dL for triglycerides, and within 0.1 % for serum HbA_1c_. For the purpose of this study, the estimated glomerular filtration rate (eGFR) was calculated using the Modification of Diet in Renal Disease equation [8].

For each participant, urine samples were collected in the morning after a 12-hour fast at the first clinic visit and after 24 weeks of pharmacologic therapy. The urinary ACR was measured by the turbidimetric method using Beckman Coulter UniCel DXC 800 Synchron™ Clinical Systems (Beckman Coulter, Brea, USA). The analytical precision for urinary ACR was within 2.3 ug/mg creatinine.

### 2.4. Outcome Measures

The primary outcome measure of this study was the change in urinary ACR after completing 24 weeks of pharmacologic treatment. The changes in serum HbA_1c_, body weight, serum creatinine level, eGFR, and systolic blood pressure were considered secondary outcome measures. 

### 2.5. Ethical Approval

This study was carried out in accordance with the World Medical Association’s Declaration of Helsinki. The study was approved by the Institutional Review Board of Changhua Christian Hospital (CCH IRB Identifier: 190512) and listed in a clinical trial registry (ClinicalTrials.gov Identifier: NCT03983551). All participants provided written informed consent to participate in the study in accordance with the Declaration of Helsinki.

### 2.6. Statistical Analysis Plan

A power analysis suggested that a sample size of 22 participants in each treatment group would be necessary to detect a significant change in urinary ACR from baseline with 80% statistical power, and the anticipated treatment effect size, expressed as the Cohen’s *d* coefficient, was 0.5. The treatment groups included all participants who received at least one dose of antidiabetic medication. The first laboratory test prior to pharmacologic intervention was considered as the baseline. Outcome measures in this study were based on laboratory data after 24 weeks of pharmacologic therapy. Participants who missed the follow up or withdrew from the study were assessed by an intention to treat analysis.

The article "Comparing the Effect of Dipeptidyl-Peptidase 4 Inhibitors and Sulfonylureas on Albuminuria in Patients with Newly Diagnosed Type 2 Diabetes Mellitus: A Prospective Open-Label Study" was published in 2019. Journal: J Clin Med.

The demographic characteristics and clinical outcomes of the treatment groups were compared using a Student’s independent *t*-test for continuous variables and Pearson’s χ^2^-test for categorical variables. A dependent *t*-test was used to compare the changes in urinary ACR, serum HbA_1c_, body weight, and serum creatinine relative to baseline levels. A statistical analysis was performed using IBM SPSS version 22.0 (IBM SPSS Statistics for Windows, New York, USA). A two-tailed *P* value of less than 0.05 indicated statistical significance. 

## 3. Results

This study screened 120 patients for eligibility. Eleven patients were excluded due to concomitant use of ACEI or ARB, and eight were ineligible because they were previously diagnosed with non-diabetic kidney disease. The enrollment process is illustrated in Figure 1.

### 3.1. Demographic Characteristics of Participants

The study enrolled 101 participants, with 45 recipients of DPP-4 inhibitors and 56 of sulfonylureas. Their demographic features are summarized in Table 1. Both treatment groups had comparable mean age (62.9 years vs. 64.3 years, *P* = 0.5), body weight (68.5 kg vs. 66.2 kg, *P* = 0.48), systolic blood pressure (134 mm Hg vs. 133 mm Hg, *P* = 0.802), and serum HbA_1c_ (8.7% vs. 8.9%, *P* = 0.66). Moreover, participants in both groups had similar mean urinary ACR at diagnosis (29.2 µg/mg creatinine vs. 39.9 µg/mg creatinine, *P* = 0.157). Similar proportions of patients in both treatment groups received antihypertensive medications including calcium channel blockers (26.7% vs. 37.5%, *P* = 0.249), beta blockers (24.4% vs. 17.8%, *P* = 0.418), and diuretics (6.7% vs. 7.1%, *P* = 0.925). Patients receiving ACEI or ARB were ineligible because these medications can modify urinary albumin excretion. All participants completed the 24-week clinical trial without loss of follow-up.

### 3.2. Comparison of the Clinical Outcomes Relative to Baseline Levels

After 24 weeks of antidiabetic therapy, urinary ACR was significantly reduced in recipients of DPP-4 inhibitors relative to baseline levels (29.2 µg/mg creatinine vs. 14.9 µg/mg creatinine, *P* < 0.001). In contrast, urinary albumin excretion was not significantly influenced by sulfonylureas relative to levels at diagnosis (39.9 µg/mg creatinine vs. 43.2 µg/mg creatinine, *P* = 0.641). Moreover, body weight was slightly reduced relative to baseline in recipients of DPP-4 inhibitors (68.5 kg vs. 67.4 kg, *P* = 0.0169) but remained unchanged in the sulfonylurea group (66.2 kg vs. 66.4 kg, *P* = 0.868). In both treatment groups, serum creatinine, eGFR, and systolic blood pressure were not significantly affected by antidiabetic therapy. These findings are recorded in Table 2.

The article "Comparing the Effect of Dipeptidyl-Peptidase 4 Inhibitors and Sulfonylureas on Albuminuria in Patients with Newly Diagnosed Type 2 Diabetes Mellitus: A Prospective Open-Label Study" was published in 2019. Journal: J Clin Med.

### 3.3. Comparison of the Clinical Outcomes between DPP-4 Inhibitors and Sulfonylureas

In terms of the primary outcome measure, participants who received DPP-4 inhibitors had a significant reduction in urinary ACR relative to recipients of sulfonylureas (−14.3 µg/mg creatinine vs. 3.29 µg/mg creatinine, *P* = 0.037). Regarding the secondary outcome measures, both groups demonstrated comparable changes in serum HbA_1c_ (−1.87 % vs. −2.40 %, *P* = 0.250), body weight (−1.04 kg vs. 0.12 kg, *P* = 0.203), serum creatinine (−0.01 mg/dL vs. 0.08 mg/dL, *P* = 0.171), eGFR (8.94 mL/min/1.73 m^2^ vs. −4.93 mL/min/1.73 m^2^, *P* = 0.104) and systolic blood pressure (−4.27 mm Hg vs. −1.14 mm Hg, *P* = 0.333) after 24 weeks of antidiabetic therapy. These findings are shown in Table 3.

## 4. Discussion

As observed in this study, DPP-4 inhibitors significantly lowered urinary albumin excretion in diabetic patients after 24 weeks of therapy. In contrast, sulfonylureas had no significant effect on urinary ACR despite their glucose-lowering capacity. Moreover, recipients of DPP-4 inhibitors demonstrated a significantly reduced body weight. Since both treatment groups attained comparable levels of serum HbA_1c_ at study completion, the effect of DPP-4 inhibitors on albuminuria may involve pathways in addition to glycemic control. 

However, this study did not detect a significant effect of either DPP-4 inhibitors or sulfonylureas on eGFR in diabetic patients. Specifically, albuminuria is often considered an early manifestation of DKD that precedes the decline in eGFR [9], and whether a reduction in albuminuria in recipients of DPP-4 inhibitors will lead to preservation of eGFR requires a longer observation time.

Several randomized clinical studies have shown that DPP-4 inhibitors may reduce albuminuria compared to placebo in patients with T2DM. In the CARMELINA study, the DPP-4 inhibitor Linagliptin attenuated albuminuria progression compared to placebo but did not have a significant effect on eGFR [10]. Similarly, in the SAVOR-TIMI study, Saxagliptin improved urinary ACR in diabetic patients without affecting their eGFR levels [11]. In a prospective clinical study, patients receiving Sitagliptin also demonstrated a significant reduction in albuminuria [12]. Overall, pharmacologic agents targeting the DPP-4 enzyme appear to have a beneficial effect on albuminuria in patients with T2DM.

The article "Comparing the Effect of Dipeptidyl-Peptidase 4 Inhibitors and Sulfonylureas on Albuminuria in Patients with Newly Diagnosed Type 2 Diabetes Mellitus: A Prospective Open-Label Study" was published in 2019. Journal: J Clin Med.

DPP-4 inhibitors may attenuate the progression of albuminuria through several mechanisms. Investigators have documented an anti-inflammatory effect of DPP-4 inhibitors that can protect renal tubular cells from damage [13]. These medications may lower oxidative stress and improve endothelial function in the kidney [14], thereby reducing the detrimental effect of chronic hyperglycemia on urinary albumin excretion. Moreover, DPP-4 inhibitors have been shown to prevent kidney fibrosis in patients with longstanding T2DM [15].

In a previous study, patients receiving sulfonylureas experienced faster deterioration of kidney function compared to recipients of metformin therapy, presumably through an increase in body mass index and systolic blood pressure [16]. Another investigation reported an increase in albuminuria in recipients of gliclazide, although the underlying mechanism remains elusive [17]. Overall, sulfonylureas may have a neutral effect on DKD due to its propensity to increase body weight and blood pressure, which counteracts the protective effect of glucose-lowering in diabetic patients. 

As shown in this clinical trial, DPP-4 inhibitors significantly lowered serum HbA_1c_ in patients with newly diagnosed T2DM. As established in previous studies, an improvement in hyperglycemia offers substantial defense against the development and progression of microalbuminuria in the diabetic kidney [18]. Furthermore, this investigation demonstrates a significant, albeit modest, effect of DPP-4 inhibitors on weight reduction. Obesity can induce glomerular hypertrophy in diabetes and accelerate the development of microalbuminuria [19]. The current study did not show an effect of this medication on blood pressure, which is another important determinant of DKD [20]. Therefore, in the context of this study DPP-inhibitors may lower albuminuria through their glucose-lowering effect and weight reduction.

The observation that DPP-4 inhibitors can reduce albuminuria in diabetic patients has clinical implications. Given the insidious course and heterogeneous presentation of DKD [21], intervention to reduce urinary albumin excretion may improve the clinical outcome. The DPP-4 inhibitor is already a favorable antidiabetic medication due to its neutral effect on body weight and relatively low risk of hypoglycemia. In addition, this study shows the beneficial effect of DPP-4 inhibitors on body weight and urinary ACR relative to sulfonylureas. Therefore, attenuation of albuminuria may be an additional consideration when selecting an antidiabetic medication.

The article "Comparing the Effect of Dipeptidyl-Peptidase 4 Inhibitors and Sulfonylureas on Albuminuria in Patients with Newly Diagnosed Type 2 Diabetes Mellitus: A Prospective Open-Label Study" was published in 2019. Journal: J Clin Med.

To our knowledge, this is the first study to directly compare DPP-4 inhibitors and sulfonylureas with the primary outcome of albuminuria reduction. This study reduces the potential confounding effect of previous antidiabetic mediations on albuminuria by enrolling patients with newly diagnosed T2DM. Moreover, participants had comparable levels of serum HbA_1c_ after antidiabetic therapy, which may lessen any confounding effect of glucose-lowering on urinary albumin excretion. Finally, recipients of ACEI or ARB were excluded due to the established effect of these medications on urinary albumin excretion. 

Nonetheless, the study design has limitations. Metformin also attenuates albuminuria by reducing oxidative stress and mesangial cell apoptosis [22]. Since all participants received metformin in addition to either DPP-4 inhibitors or sulfonylureas, a beneficial effect of metformin on urinary ACR becomes a potential confounding factor. Moreover, epidemiological evidence has suggested a strong genetic basis for DKD [23], but a family history of kidney disease was not accounted for in this study. Previous investigators have proposed that since hyperglycemia can accelerate urinary albumin excretion [24], the influence of antidiabetic medications on albuminuria may still partly depend on their glucose-lowering capacity. Finally, the non-randomized design and relatively small sample size may limit the robustness of this study. Randomized studies with a larger sample size will be necessary to confirm the findings of this investigation.

## 5. Conclusions

In conclusion, the addition of DPP-4 inhibitors to metformin therapy in patients with T2DM significantly reduced urinary albumin excretion relative to recipients of sulfonylureas. Importantly, the beneficial effect of DPP-4 inhibitors occurred despite attaining similar levels of glycemic control as sulfonylureas. Overall, DPP-4 inhibitors may have a role in attenuating the progression of albuminuria, and albuminuria reduction may be an additional consideration when choosing between antidiabetic medications.

## Figures and Tables

**Figure 1:** Enrollment protocol of the study. ACEI: angiotensin-converting enzyme inhibitors, ARB: angiotensin receptor blockers.

**Table 1:** Demographic features of participants at diagnosis of type 2 diabetes mellitus.

Variables	DPP-4 Inhibitors + Metformin (*n* = 45)	Sulfonylureas + Metformin (*n* = 56)	*P* Value
Age (years)	62.9 ± 14.0	64.3 ± 10.7	0.500
Sex (Female)	22 (52.4%)	25 (47.2%)	0.682
Body weight (kg)	68.5 ± 16.0	66.2 ± 15.1	0.48
Serum HbA_1c_ (%)	8.7 ± 1.9	8.9 ± 1.8	0.66
Creatinine (mg/dL)	0.83 ± 0.19	0.86 ± 0.25	0.379
Estimated GFR (mL/min/1.73 m^2^)	88.5 ± 24.8	89.6 ± 26.7	0.843
ALT (U/mL)	33.0 ± 29.5	28.8 ± 22.1	0.430
Systolic blood pressure (mm Hg)	134 ± 19.4	133 ± 14.8	0.802
Urinary ACR (µg/mg creatinine)	29.2 ± 31.2	39.9 ± 41.9	0.157
Triglycerides (mg/dL)	162 ± 118	189 ± 116	0.278
High density lipoprotein cholesterol (mg/dL)	44.2 ± 12.3	46.3 ± 14.3	0.455
Low density lipoprotein cholesterol (mg/dL)	110 ± 34.8	117 ± 32.7	0.277
Use of calcium channel blockers	12 (26.7%)	21 (37.5%)	0.249
Use of beta blockers	11 (24.4%)	10 (17.8%)	0.418
Use of diuretics	3 (6.7%)	4 (7.1%)	0.925

Data are expressed as means with a standard deviation of the mean for continuous variables and number (%) for categorical variables. Variables are compared between groups using Student’s *t*-test for continuous data. ALT: alanine aminotransferase, HbA_1c_: glycosylated hemoglobin A_1c_, ACR: albumin-to-creatinine ratio, DPP-4: dipeptidyl-peptidase 4, GFR: glomerular filtration rate.

The article "Comparing the Effect of Dipeptidyl-Peptidase 4 Inhibitors and Sulfonylureas on Albuminuria in Patients with Newly Diagnosed Type 2 Diabetes Mellitus: A Prospective Open-Label Study" was published in 2019. Journal: J Clin Med.

**Table 2:** Comparison of outcome measures relative to levels at diagnosis.

Treatment Duration	DPP-4 Inhibitors + Metformin (*n* = 45)	Sulfonylureas + Metformin (*n* = 56)
Urinary ACR (µg/mg creatinine)		
0 week	29.2 ± 31.2	39.9 ± 41.9
24 weeks	14.9 ± 23.9	43.2 ± 64.2
*P* value	< 0.001	0.641
Serum HbA_1c_ (%)		
0 week	8.7 ± 1.9	8.9 ± 1.8
24 weeks	6.8 ± 0.83	7.2 ± 1.0
*P* value	<0.001	<0.001
Body weight (kg)		
0 week	68.5 ± 16.0	66.2 ± 15.1
24 weeks	67.4 ± 15.8	66.4 ±14.4
*P* value	0.0169	0.868
Serum creatinine (mg/dL)		
0 week	0.83 ± 0.19	0.86 ± 0.24
24 weeks	0.85 ± 0.28	0.95 ± 0.35
*P* value	0.846	0.058
Estimated GFR (mL/min/1.73 m^2^)		
0 week	88.5 ± 24.8	89.6 ± 26.7
24 weeks	97.5 ± 47.5	84.6 ± 30.3
*P* value	0.233	0.225
Systolic blood pressure (mm Hg)		
0 week	134 ± 19.4	133 ± 14.8
24 weeks	128 ± 13.2	131 ± 10.6
*P* value	0.113	0.56

Data are expressed as means with a standard deviation of the mean for continuous variables. Variables are compared to baseline levels using the paired *t*-test. HbA_1c_: glycosylated hemoglobin A_1c_, ACR: albumin-to-creatinine ratio, kg: kilograms, mg/dL: milligrams per deciliter, mm Hg: millimeters of mercury, DPP-4: dipeptidyl-peptidase 4, GFR: glomerular filtration rate.

**Table 3:** Comparison of outcome measures between dipeptidyl-peptidase 4 inhibitors and sulfonylureas.

Treatment Duration	DPP-4 Inhibitors + Metformin (*n* = 45)	Sulfonylureas + Metformin (*n* = 56)	*P* Value
Change in urinary ACR (µg/mg creatinine)			
24 weeks	−14.3 ± 21.2	3.29 ± 52.5	0.037
Change in serum HbA_1c_ (%)			
24 weeks	−1.87 ± 2.00	−2.40 ± 2.43	0.250
Change in body weight (kg)			
24 weeks	−1.04 ± 2.82	0.12 ± 5.55	0.203
Change in serum creatinine (mg/dL)			
24 weeks	−0.01± 0.359	0.08 ± 0.32	0.171
Change in estimated GFR (mL/min/1.73 m^2^)			
24 weeks	8.94 ± 49.6	−4.93 ± 30.0	0.104
Change in systolic blood pressure (mm Hg)			
24 weeks	−4.27 ± 17.7	−1.14 ± 14.6	0.333

Data are expressed as means with a standard deviation of the mean for continuous variables. Variables are compared between groups using Student’s *t*-test. HbA_1c_: glycosylated hemoglobin A_1c_, ACR: albumin-to-creatinine ratio, kg: kilograms, mg/dL: milligrams per deciliter, mm Hg: millimeters of mercury, DPP-4: dipeptidyl-peptidase 4, GFR: glomerular filtration rate.
